The article "Cytoprotective Effect of Benzyl N'-(5-Chloro-indol-3-yl-methylidene)-hydrazinecarbodithioate Against Ethanol-Induced Gastric Mucosal Injury in Rats" was retracted in 2013. Reasons: duplicated data; duplicate publication; concerns about the data.

# Cytoprotective Effect of Benzyl *N'*-(5-Chloro-indol-3-yl-methylidene)-hydrazinecarbodithioate Against Ethanol-Induced Gastric Mucosal Injury in Rats

**DOI:** 10.3390/molecules17089306

**Published:** 2012-08-03

**Authors:** Harita Hashim, Fathi F. Mughrabi, Mahmood Ameen, Hamid Khaledi, Hapipah M. Ali

**Affiliations:** 1 Department of Biology, Faculty of Applied Science, University Teknologi MARA, Shah Alam 40450, Malaysia; 2 Department of Zoology, Faculty of Science, University of Benghazi, P.O. Box 18019, Benghazi, Libya; 3 Department of Molecular Medicine, Faculty of Medicine, University of Malaya, Kuala Lumpur 50603, Malaysia; 4 Department of Chemistry, Faculty of Science, University of Malaya, Kuala Lumpur 50603, Malaysia

**Keywords:** indole, benzyl *N'*-(5-chloroindol-3-ylmethylidene)hydrazinecarbodithioate, histology, omeprazole, gastric ulcer

## Abstract

Indolic compounds have attracted a lot of attention due to their interesting biological properties. The present study was performed to evaluate the subacute toxicity and anti-ulcer activity of BClHC against ethanol-induced gastric ulcers. Experimental animal groups were orally pre-treated with different doses of BClHC (50, 100, 200 and 400 mg/kg) in 10% Tween 20 solution (vehicle). Blank and ulcer control groups were pre-treated with vehicle. The positive group was orally pretreated with 20 mg/kg omeprazole. After one hour, all groups received absolute ethanol (5 mL/kg) to generate gastric mucosal injury except the blank control group which was administered the vehicle solution. After an additional hour, all rats were sacrificed, and the ulcer areas of the gastric walls determined. Grossly, the ulcer control group exhibited severe mucosal injury, whereas pre-treatment with either derivative or omeprazole resulted in significant protection of gastric mucosal injury. Flattening of gastric mucosal folds was also observed in rats pretreated with BClHC. Histological studies of the gastric wall of ulcer control group revealed severe damage of gastric mucosa, along with edema and leucocytes infiltration of the submucosal layer compared to rats pre-treated with either BClHC or omeprazole where there were marked gastric protection along with reduction or absence of edema and leucocytes infiltration of the submucosal layer. Subacute toxicity study with a higher dose of derivative (5 g/kg) did not manifest any toxicological signs in rats. In conclusions, the present finding suggests that benzyl *N'*-(5-chloroindol-3-ylmethylidene)hydrazinecarbodithioate promotes ulcer protection as ascertained by the comparative decreases in ulcer areas, reduction of edema and leucocytes infiltration of the submucosal layer.

## 1. Introduction

Indolic compounds have attracted a lot of attention due to their interesting biological properties. Antioxidant [1,2], anticancer [3,4], antiviral [5], antiulcer [6] and wound healing activities [7] can be mentioned as some of the significant activities associated with the indole nucleus. Likewise, derivatives of dithiocarbazic acid have been proven to exhibit a wide variety of bioactivities such as antimicrobial [8], anticancer [9], antibacterial and antifungal [10] properties. Through our ongoing efforts to develop new potent wound healing agents, we recently reported the wound healing potential of the Schiff base formed from indole-3-carboxaldehyde and S-benzyldithiocarbazate [11]. The present findings suggest that BClHC promotes ulcer protection as ascertained grossly by significant reduction of ulcer area, and histologically by comparative decreases in ulcer areas, reduction or absence of edema and leucocytes infiltration of the submucosal layer compared to the ulcer control group.

## 2. Results and Discussion

### 2.1. Subacute Toxicity

Study in which the animals were treated with doses of 2 and 5 g/kg of BClHC did not manifest any significant abnormal signs and behavioral changes. There was no mortality with these oral doses at the end of 14 days of observation (Figure 1). The serum biochemistry parameters (liver function tests) of the BClHC treated rats showed no significant changes compared to the control normal rats. From these results it is concluded that this compound has no subacute toxicity and the oral lethal dose for the male and female rats is in excess of 5 g/kg of BClHC (Table 1 and Table 2).

**Figure 1:** Histological sections of liver and kidney in subacute toxicity test (**A**) liver of rats treated with vehicle (10% Tween 20, 5 mL/kg) showing normal structural appearance; (**B**) kidney of rats treated with vehicle (10% Tween 20, 5 mL/kg) showing normal structural appearance; (**C**) Liver of rats treated with 2 g/kg of BClHC showing normal structural appearance; (**D**) Kidney of rats treated with 2 g/kg of BClHC showing normal structural appearance; (**E**) Liver of rats treated with 5 g/kg of BClHC showing normal structural appearance; (**F**) kidney of rats treated with 5 g/kg of BClHC showing normal structural appearance.

**Table 1:** Renal function test of rats in acute toxicity study of BClHC compound.

Animal Groups	Renal Function Test of BClHC						
	Sodium (mmol/L)	Pottasium (mmol/L)	Chloride (mmol/L)	CO_2_ (mmol/L)	Anion gap (mmol/L)	Urea (mmol/L)	Creatinine (µmol/L)
**Normal** ** control**	138.34 ± 0.62	5.12 ± 0.17	103.42 ± 0.76	22.70 ± 0.73	19.34 ± 0.76	5.68 ± 0.36	50.78 ± 1.30
**L. D** ** (2 g/kg)**	138.42 ± 0.74	5.25 ± 0.18	102.67 ± 1.06	20.63 ± 0.69	19.67 ± 1.08	5.19± 0.34	49.12 ± 0.85
**H. D** ** (5 g/kg)**	138.29 ± 0.67	4.94 ± 0.20	102.50 ± 0.70	22.29 ± 0.72	18.58 ± 0.61	5.78 ± 0.30	49.25 ± 1.39

Values expressed as means ± S.E.M. There are no significant differences between groups. Significant values at *p* < 0.05.

**Table 2:** Liver function test of rats in acute toxicity study of **BClHC** compound.

Animal Groups	Liver Function test of BClHC								
	Total protein (g/L)	Albumin (g/L)	Globulin (g/L)	Total bilirubin (µmol/L)	Conjugated bilirubin (µmol/L)	AP (IU/L)	ALT (IU/L)	AST (IU/L)	G-Glutaml. Transferase (IU/L)
**Normal** ** control**	70.34 ± 1.25	11.58 ± 0.63	59.17 ± 1.23	2.04 ± 0.20	1.25 ± 0.25	135.08 ± 9.27	53.00 ± 1.97	152.31 ± 5.14	4.96 ± 0.71
**L.D** ** (2 g/kg)**	70.25 ± 0.85	11.92 ± 0.41	58.59 ± 0.51	2.21 ± 0.20	1.42 ± 0.16	134.17 ± 4.77	50.92 ± 1.12	157.59 ± 2.11	4.88 ± 0.85
**H D** ** (5 g/kg)**	70.42 ± 0.94	12.17 ± 0.68	58.67 ± 0.85	1.82 ± 0.23	1.59 ± 0.06	135.08 ± 3.86	51.84 ± 3.57	153.84 ± 6.64	5.33 ± 0.71

Values expressed as mean ± S.E.M. There are no significant differences between groups. Significant value at *p* < 0.05; T. Prot: Total protein; TB: Total bilirubin; CB: Conjugated bilirubin; AP: Alkaline phosphatase; ALT: Alanine aminotransferase; AST: Aspartate aminotransferase; AG: anion gap; Crt: creatinine.

### 2.2. Gross Evaluation of Gastric Lesions

Rats pre-treated with either omeprazole or various concentrations of BClHC before being given absolute alcohol had significantly reduced areas of gastric ulcer formation compared to rats pre-treated with vehicle, 10% Tween 20 solution (ulcer group) (Table 3 and Figure 2). Moreover, BClHC administration significantly suppressed the formation of the ulcers and it was interesting to note the flattening of gastric mucosal folds in rats pretreated with this compound. It was also observed that protection of gastric mucosa was more prominent in rats pre-treated with 400 mg/kg BClHC (Table 3). In addition, ethanol-induced mucosal damage was significantly and dose-dependently reduced in size and severity by pre-treating the animals with BClHC (the significant inhibition of gastric ulcers in pretreatment with BClHC was compared with omeprazole, which is a standard drug used for curing gastric ulcers).

**Table 3:** Observed ulcer area and inhibition percentage of **BClHC** in rats.Values are means ± SEM of six animals.

Group	Pretreatment 5 mL/Kg	Ulcer (mm^2^) X ± SEM	Inhibition %
1	10% Tween 20	922.00 ± 7.63 **^a^**	0.00
2	Omeprazole	215.00 ± 4.54 **^b^**	76.68%
3	50 mg/Kg	54.00 ± 3.08 **^c^**	94.14%
4	100 mg/Kg	38.40 ± 2.400 **^cd^**	95.84%
5	200 mg/Kg	22.80 ± 2.89 **^de^**	97.53%
6	400 mg/Kg	12.00 ± 2.400 **^ef^**	98.70%

All values are expressed as means ± standard error mean. Means with different superscripts are significantly different. The mean difference is significant at the *p* < 0.05 level.

**Figure 2:** Gross appearance of the gastric mucosa in rat, (**A**) pre-treated with vehicle 0.2 mL of 10% Tween 20 (ulcer control). Severe injuries are seen in the gastric mucosa (arrow).Absolute ethanol produced extensive visible hemorrhagic necrosis of gastric mucosa; (**B**) Rats pre-treated with omeprazole (20 mg/Kg). Injuries to the gastric mucosa are milder (arrow) compared to the injuries seen in the ulcer control rats; (**C**) Rats pre-treated with BClHC (100 mg/Kg). Mild injuries to the gastric mucosa can be seen showing the beginning of gastric mucosa flattening; (**D**) Rats pre-treated with BClHC (200 mg/Kg). Very mild injuries to the gastric mucosa can be seen, showing the flattening of gastric mucosa, (**E**) Rats pre-treated with BClHC alone (400 mg/Kg). No injuries to the gastric mucosa are seen, but the flattening of gastric mucosa can been seen.

### 2.3. Histological Evaluation of Gastric Lesions

Microscopic observations of ethanol-induced gastric lesions in ulcer control rats (pre-treated with vehicle, 10% Tween 20), showed marked extensive damage to the gastric mucosa, and edema and leucocytes infiltration of the submucosal layer (Figure 3A). Rats that were pre-treated with either BClHC or omeprazole each had comparatively better protection of the gastric mucosa as seen by the reduction in ulcer area, reduced submucosal edema and absence of leucocytes infiltration (Figure 3B,C). The BClHC has been shown to exert the cytoprotective effects in a dose-dependent manner.

**Figure 3:** Histological sections of the ethanol-induced gastric mucosal damage in rats (H&E stain 10×). (**A**) Rats pre-treated with 5 mL/Kg of 10% Tween 20 solution (ulcer control). There is severe disruption to the surface epithelium, and edema of the submucosal layer with leucocytes infiltration. (**B**) Rats pre-treated with 20 mg/kg of omeprazole. There is mild disruption to the surface epithelium with no edema and no leucocytes infiltration of the submucosal layer. (**C**) Rats pre-treated with 200 mg/kg of BClHC. There is very mild disruption to the surface epithelium with no edema and no leucocytes infiltration of the submucosal layer. (**D**) Rats pre-treated with 400 mg/kg of BClHC. There is no disruption to the surface epithelium with the absence of edema and leucocytes infiltration of the submucosal layer.

### 2.4. Periodic Acid Schiff (PAS) of Mucosal Glycoprotein’s

Increased the PAS staining (magenta color) of gastric mucosa of treated animals with BClHC comparison to ulcer control group indicating increase in glycoprotein content of gastric mucosa. BClHC-treated group reserved the decrease in PAS staining induced by ethanol (Figure 4).

**Figure 4:** The effect of BClHC on gastric tissue glycoprotein-PAS staining in ethanol-induced gastric ulcer in rats(PAS stain 20×). (**A**) Normal control group; (**B**) Ulcer control group; (**C**) BClHC-treated group with 50 mg/kg; (**D**) BClHC-treated group with 400 mg/kg.

This study investigated the effects of BClHC on gastric ulcer compared to omeprazole, a drug whose ulcer healing effects have been extensively studied. The present compound (BClHC) is a hybrid molecule, obtained by condensation of two pharmacophores: indole carbaldehyde and S-benzyl-dithiocarbazate. Schiff bases derived by condensation of heterocyclic aldehydes with S-benzyl-dithiocarbazate have been shown to exhibit significant biological activities. It has been proposed that the biological activity of these Schiff bases may come from their interaction with potential donors of biological heterocyclic *in* *vivo*. In many cases, the pharmacological activity has been found to be highly dependent on the identity of the donor sequence of the ligands, as different ligands show widely different biological activities, although they may vary only slightly in their molecular structure. 

BClHC was found to have a protective effect on the gastric mucosa similar to that of omeprazole. Omeprazole and BClHC were both found to have protective effects compared to the ulcer control group (10% Tween 20). This suggests that BClHC does indeed have a potential anti-ulcer effect. 

BClHC has been shown to display anti-cancer activity [9] and it is speculated that the gastro-protective effect exerted by BClHC could be attributed to this anti-cancer activity, which could also be a key factor in the prevention of gastric ulcer as reported by Das and Livingstone [12].

Microbial infection of wounds delays healing [13] and causes a more pronounced subacute inflammatory reactions [14], which can lead to further tissue injury and damage. It is also important to mention that BCIHC has demonstrated an antimicrobial activity [8], that may partly contribute to the wound healing effect by eliminating infections, thus allowing the natural tissue repair processes to start. It also suggests that the BCIHC may also play a useful role in accelerating the healing of old wounds by eradicating already established infections. The antimicrobial activity of honey and the essential oil of *Melaleuca alternifolia* are believed to underlie their usefulness as alternative therapy in wound healing [15,16].

The main cause of gastric ulcer is destruction of the gastric mucosal barrier consisting of the surface epithelium and mucosal coat. This destruction may be due to an increase in gastric acid secretion, decrease in mucus production or decrease in mucosal blood flow [17]. Ethanol administration is a simple method used for inducing gastric ulcers in experimental rats and leads to severe gastric mucosal injury. Ethanol shows its harmful effects either through direct generation of reactive metabolites, including free radical species that react with most of the cell components, changing their structures and functions, or promote enhanced oxidative damage [18,19]. Ethanol damage to the gastrointestinal mucosa with microvascular injury, disruption of the vascular endothelium resulting in increased vascular permeability, edema formation and epithelial lifting [20]. It produces necrotic lesions in the gastric mucosa by its direct toxic effect, reducing the secretion of bicarbonates and production of mucus [21]. Ethanol is metabolized in the body releasing superoxide an ion and hydroperoxyl free radicals which are involved in the mechanism of subacute and chronic ulceration in the gastric mucosa [22]. Observed that administration of ethanol caused disturbances in gastric secretion, damage to the gastric mucosa, alterations in permeability, gastric mucus depletion and free-radical production. 

Oxidative stress plays a major role in the pathogenesis of various diseases including gastric ulcer. Indolic compounds have shown to possess antioxidant activity [23,24] which may mediate the protection of gastric mucosa. Antioxidants are important inhibitors of lipid per-oxidation, not only for food protection but also as a defense mechanism of living cells against oxidative damage [25]. Antioxidants have been reported to play a significant role in preventing gastric ulcers. It appears that antioxidant may be an important contributory factor in the protection of gastric mucosa [26]. Studies have shown that antioxidant significantly strength gastric walls and protect tissues from oxidative damage [27]. The result of the present study also revealed protection of gastric mucosa and inhibition of leucocytes infiltration of gastric wall in rats pretreated with BClHC. Similarly, Kobayashi *et al*. [28] reported that teprenone exerts a protective effect against mucosal lesions through inhibition of neutrophil infiltration in the ulcerated gastric tissue and [29] demonstrated that the reduction of neutrophil infiltration into ulcerated gastric tissue promotes the healing of gastric ulcers in rats [30], showed that oral administration of compound before ethanol administration significantly decreased neutrophil infiltration of gastric mucosa. Absolute alcohol would extensively damage the gastric mucosa leading to increased neutrophil infiltration into the gastric mucosa. Oxygen free radicals derived from infiltrated neutrophils in ulcerated gastric tissues have inhibitory effect on gastric ulcers healing in rats [31]. Neutrophils mediate lipid per-oxidation through the production of superoxide anions [32]. Neutrophils are a major source of inflammatory mediators and can release potent reactive oxygen species such as superoxide, hydrogen peroxide and myeloperoxidase derived oxidants. These reactive oxygen species are highly cytotoxic and can induce tissue damage [30]. Furthermore, neutrophil accumulation in gastric mucosa has been shown to induce microcirculatory abnormalities [33]. Suppression of neutrophils infiltration during inflammation was found to enhance gastric ulcer healing [34].

In the current study, we observed flattening of the mucosal folds, which suggests that the gastroprotective effect of BClHC might be due to a decrease in gastric motility. It is reported that changes in the gastric motility may play a role in the development and prevention of experimental gastric lesions [35,36]. Relaxation of circular muscles may protect the gastric mucosa through flattening of the folds. This will increase the mucosal area exposed to necrotizing agents and reduce the volume of the gastric irritants on regal crest [37]. Ethanol produces a marked contraction of the circular muscles of rat fundic strip, and such a contraction can lead to mucosal compression at the site of the greatest mechanical stress, at the crests of mucosal folds leading to necrosis and ulceration [38].

The subacute toxicity profile of BClHC could be considered favorable, judging for the absence of adverse clinical manifestations in experimental animals after two week of observation. It is concluded that subacute toxicity study with a higher dose of BClHC (5 g/kg) did not manifest any toxicological signs in rats and that the oral lethal dose for male and female albinos Wistar rats is in excess of 5 g/kg. Based on this subacute toxicity test, BClHC was found safe. In conclusion, BClHC could significantly protect the gastric mucosa against ethanol-induced injury. Such protection was shown to be dose dependent as ascertained by the reduction or inhibition of ulcer areas in the gastric wall as well as the reduction or inhibition of edema and leucocytes infiltration of submucosal layers, and protection was most prominent at a dose of 400 mg/kg BClHC.

## 3. Experimental

### 3.1. Omeprazole

Omeprazole is a proton pump inhibitor which has been widely used as acid inhibitor agents for the treatment of disorders related to gastric acid secretion for the last 15 years [39]. Omeprazole is a substituted benzimidazole that inhibits acid secretion by acting on the hydrogen-potassium exchanger (H^+^/K^+^-ATPase) for the apical plasma membrane of the gastric mucosa [40]. Omeprazole is highly selective for the proton pump and undergo catalyzed conversion into active form within the acid forming space. The active inhibitors react with SH (thiol) group of the proton pump, resulting in inhibition of acid formation [41]. In this study, omeprazole was used as the reference anti-ulcer drug, and was obtained from the University Malaya Medical Centre (UMMC) Pharmacy. The drug was dissolved in 10% Tween 20 solution and administered orally to the rats in doses of 20 mg/kg body weight (5 mL/kg) [42].

### 3.2. Synthesis of Benzyl N'-(5-Chloro-indol-3-ylmethylidene)hydrazinecarbodithioate

S-benzyldithiocarbazate was prepared as reported previously [43]. Briefly, 5-chloroindole-3-carbaldehyde (5.39 g, 0.03 mol) and *S*-benzyl dithiocarbazate (5.94 g, 0.03 mol) were heated in ethanol (300 mL) for 3 h. The solution was set aside for few hours whereupon a yellow precipitate formed. This precipitate was filtered off, washed with cold ethanol and dried over silica gel; yield, 9.8 g (91%) (Figure 5). 

**Figure 5:** Benzyl *N'*-(5-chloroindol-3-ylmethylidene)hydrazinecarbodithioate.

### 3.3. Experimental Animals

Adult male albino Wistar rats were obtained from the Animal House, Faculty of Medicine, University of Malaya, Kuala Lumpur, Malaysia. All the animals used for study has an ethical clearance from the animal user’s Committee of the Faculty of Medicine, University Malay (Ethics No. PM 28/9/2008 MAA (R)). The rats weighed between 200–220 g. They were fasted for 48 hours before the experiment [44], but were allowed free access drinking water until 2 hours before the experiment. During the fasting period, the rats were placed individually in separate cages with wide-mesh wire bottoms. On the day of the experiment, the rats were randomly divided into seven groups of six rats each. Throughout the experiments, all animals received human care according to the criteria outlined in the “Guide for the Care and Use of Laboratory Animals” prepared by the National Academy of Sciences and published by the U.S. National Institutes of Health [45].

### 3.4. Subacute Toxicity Studies

The subacute toxic study was used to determine a safe dose for the BClHC. Thirty six albino Wistar rats (18 males and 18 females) were assigned equally into three groups labeled as vehicle (10% Tween 20); 2 g/kg and 5 g/kg of BClHC in vehicle preparation, respectively. The animals were fasted overnight (food but not water) prior to dosing. Food was withheld for a further 3 to 4 hours after dosing. The animals were observed for 30 min and 2, 4, 24 and 48 hours after the administration for the onset of clinical or toxicological symptoms. Mortality, if any, was observed over a period of 2 weeks. The animals were sacrificed on the 15th day. Hematological, serum biochemical and histological (liver and kidney) parameters were determined following standard methods [46,47].

### 3.5. Treatment

Gastric ulcer was induced in adult male Wistar rats by orogastric intubation of absolute ethanol (5 mL/kg) according to the method described by De Pasquale *et al*. [48] with slight modifications. Blank and ulcer control groups were orally administered with vehicle (10% Tween 20) solution. Experimental groups were orally administered with. 50, 100, 200 and 400 mg/kg of BClHC in vehicle solution (5 mL/kg), respectively. The positive group received oral doses of 20 mg/kg omeprazole in vehicle solution (5 mL/kg) as positive controls one hour after this pre-treatment; all groups of rats were gavaged with absolute ethanol (5 mL/kg) in order to induce gastric ulcers except the blank control group which was only administered vehicle solution (5 mL/kg). The rats were euthanized by cervical dislocation 60 minutes later [49] under an overdose of diethyl ether anesthesia and their stomachs were immediately excised.

### 3.6. Gross Gastric Lesions Evaluation

Any ulcers would have be found in the gastric mucosa, appearing as elongated bands of hemorrhagic lesions parallel to the long axis of the stomach. Each gastric mucosa was thus examined for damage. The length (mm) and width (mm) of the ulcer on the gastric mucosa were measured by a planimeter (10 × 10 mm^2^ = ulcer area) under dissecting microscope (×1.8). The area of each ulcer lesion was measured by counting the number of small squares, 2 mm × 2 mm, covering the length and width of each ulcer band. The sum of the areas of all lesions for each stomach was applied in the calculation of the ulcer area (UA) wherein the sum of small squares × 4 × 1.8 = UA mm^2^ as described by Kauffman and Grossman [50] with slight modifications. The inhibition percentage (I%) was calculated using a slightly modified version of the formula described by Njar *et al.* [51]:



### 3.7. Histological Evaluation of Gastric Lesions

Specimens of the gastric walls from each rat were fixed in 10% buffered formalin and processed in a paraffin tissue processing machine. Sections of the stomach were made at a thickness of 5 µm and stained with hematoxylin and eosin for histological evaluation [52].

### 3.8. Study of Mucosal Glycoproteins

Sections of 5 µm thickness of the glandular portion of the rat stomach of each group were stained with periodic acid Schiff (PAS) stain to observed mucus production and to note the changes in both acidic and basic glycoproteins [53].

### 3.9. Statistical Analysis

All values were reported as means ± S.E.M. The statistical significance of differences between groups was assessed using one-way ANOVA. A value of *p* < 0.05 was considered significant.

## 4. Conclusion

BClHC could significantly protect the gastric mucosa against ethanol-induced injury. Such protection was shown to be dose dependent as ascertained by the reduction or inhibition of ulcer areas in the gastric wall as well as the reduction or inhibition of edema and leucocytes infiltration of submucosal layers, and protection was most prominent at a dose of 400 mg/kg BClHC.
